The article "Comprehensive Analysis of Ferroptosis-Related LncRNAs in Breast Cancer Patients Reveals Prognostic Value and Relationship With Tumor Immune Microenvironment" was published in 2021. Journal: Front Surg.

# Comprehensive Analysis of Ferroptosis-Related LncRNAs in Breast Cancer Patients Reveals Prognostic Value and Relationship With Tumor Immune Microenvironment

**DOI:** 10.3389/fsurg.2021.742360

**Published:** 2021-10-04

**Authors:** Zhengjie Xu, Suxiao Jiang, Juan Ma, Desheng Tang, Changsheng Yan, Kun Fang

**Affiliations:** ^1^Department of Surgery, Yinchuan Maternal and Child Health Hospital, Yinchuan, China; ^2^Department of Ultrasound, Yinchuan Maternal and Child Health Hospital, Yinchuan, China; ^3^Department of Surgical Oncology, The First Affiliated Hospital of Harbin Medical University, Harbin, China

**Keywords:** breast cancer, ferroptosis, lncRNA, prognosis, immune microenvironment

## Abstract

**Background:** Breast cancer (BC) is a heterogeneous malignant tumor, leading to the second major cause of female mortality. This study aimed to establish an in-depth relationship between ferroptosis-related LncRNA (FRlncRNA) and the prognosis as well as immune microenvironment of the patients with BC.

**Methods:** We downloaded and integrated the gene expression data and the clinical information of the patients with BC from The Cancer Genome Atlas (TCGA) database. The co-expression network analysis and univariate Cox regression analysis were performed to screen out the FRlncRNAs related to prognosis. A cluster analysis was adopted to explore the difference of immune microenvironment between the clusters. Furthermore, we determined the optimal survival-related FRLncRNAs for final signature by LASSO Cox regression analysis. Afterward, we constructed and validated the prediction models, which were further tested in different subgroups.

**Results:** A total of 31 FRLncRNAs were filtrated as prognostic biomarkers. Two clusters were determined, and C1 showed better prognosis and higher infiltration level of immune cells, such as B cells naive, plasma cells, T cells CD8, and T cells CD4 memory activated. However, there were no significantly different clinical characters between the clusters. Gene Set Enrichment Analysis (GSEA) revealed that some metabolism-related pathways and immune-associated pathways were exposed. In addition, 12 FRLncRNAs were determined by LASSO analysis and used to construct a prognostic signature. In both the training and testing sets, patients in the high-risk group had a worse survival than the low-risk patients. The area under the curves (AUCs) of receiver operator characteristic (ROC) curves were about 0.700, showing positive prognostic capacity. More notably, through the comprehensive analysis of heatmap, we regarded LINC01871, LINC02384, LIPE-AS1, and HSD11B1-AS1 as protective LncRNAs, while LINC00393, AC121247.2, AC010655.2, LINC01419, PTPRD-AS1, AC099329.2, OTUD6B-AS1, and LINC02266 were classified as risk LncRNAs. At the same time, the patients in the low-risk groups were more likely to be assigned to C1 and had a higher immune score, which were consistent with a better prognosis.

**Conclusion:** Our research indicated that the ferroptosis-related prognostic signature could be used as novel biomarkers for predicting the prognosis of BC. The differences in the immune microenvironment exhibited by BC patients with different risks and clusters suggested that there may be a complementary synergistic effect between ferroptosis and immunotherapy.

## Introduction

Breast cancer (BC) is the most common cancer among women in the world, leading to the second largest cause of female mortality, and its morbidity and mortality are increasing year by year (1). Due to the large population base in China, the number of cases and deaths of female BC in China ranks first in the world (2). Although with the development of people's awareness of physical examination and prevention and the all-out support of diversified treatment methods, such as surgery, radiotherapy, the prognosis of BC has been significantly improved. However, the prognosis of advanced BC is still disappointing (3, 4). According to the previous research, BC is a malignant solid tumor formed by the long-term action of multiple genes and factors, accompanied by obvious heterogeneity, resulting in a diversified tumor microenvironment and different responses (5, 6). Increasing evidence showed that lncRNA plays a unignorable role in regulating the occurrence and development of various cancers, such as BC (7), endometrial cancer (8), and liver cancer (9). Therefore, we need to explore the potential molecular mechanisms to maximize the benefits of existing methods to promote the progress in the diagnosis and treatment of BC.

Ferroptosis is an iron-dependent, novel programmed cell death pattern distinct from apoptosis, cell necrosis, and autophagy that can be triggered by acute and chronic cellular stress caused by abnormal lipid metabolism and biochemical processes (10–12). The previous studies have proved that the activation of ferroptosis can promote the killing effect of body on tumors, especially for tumors that have developed resistance to the traditional treatments, such as BC, which has become a very promising anti-tumor direction (13–15). Glutathione peroxidase 4 (GPX4) can be used by BC to gain the ability to endure drug resistance, conversely, the loss of GPX4 function can reverse the formation of BC drug resistance, which leads to the persistent ferroptosis process of cells and prevents tumor recurrence, suggesting that targeting GPX4 is a therapeutic strategy for acquired drug resistance (13). In addition, siramesine combined with lapatinib promotes the death of BC cells by increasing reactive oxygen species (ROS) through iron transport disruption, independent of downstream targets (members of the EGFR family) and cathepsin B, which suggests that the other targets of siramesine and lapatinib are associated with ferroptosis and provides hope for overcoming apoptotic resistance in BC (16). In addition to GPX4, a previous study reported that other ferroptosis-related genes, such as iron, ACSL4, SLC7A11, and SLC3A, could be promising targets for BC treatment (17, 18). However, there are few studies on ferroptosis and immune microenvironment of BC, and unified insights are still lacking but urgently needed.

In the present study, we downloaded and integrated the gene expression data and the clinical information of patients with BC from the TCGA dataset. The cluster analysis was then adopted to explore the difference of immune microenvironment. Afterward, the prognostic signature associated with ferroptosis was determined to construct the predicting models and further validated these models. Collectively, not only did our results demonstrate that the prognostic models accurately predicted the prognosis of patients with BC, but also preliminarily revealed the differences in the immune microenvironment in the process of ferroptosis, which provided some thoughts and insights for the combination of immunotherapy and ferroptosis in clinical diagnosis and treatment of BC.

## Materials and Methods

### Data Collection and Process

The gene expression data of the transcriptome (such as, mRNA and LncRNA) and the clinical information of BC patients were downloaded from the TCGA dataset (19), of which the clinical information included the survival time, survival status, age, gender, grade, stage, T stage, N stage, and M stage. Specifically, we preliminarily screened 1,178 cases of transcriptome data, such as 112 cases of the normal and 1,066 cases of the tumor, and 1,053 cases of clinical data that include 911 cases of survival and 142 cases of death. A list of ferroptosis-related genes was extracted from FerrDb (http://www.zhounan.org/ferrdb/operations/download.html), and the expression of ferroptosis-related genes was extracted.

### Screening of the Prognostic FRLncRNAs

For picking out the target ferroptosis-related LncRNAs (FRlncRNAs), a co-expression network analysis was adopted to show the relationship between lncRNAs and ferroptosis-related genes. The LncRNAs with |r| ≥ 0.5 and *P* < 0.001 were confirmed as FRlncRNAs. Then, the univariate Cox regression analysis was used to screen the prognosis-related FRlncRNAs, and the results were presented in the form of forest plot. Further, we drew a heatmap and compared the differential expression of these FRlncRNAs in normal tissues and tumor tissues using the rank sum test.

### Hierarchical Consensus Clustering Based on the Prognostic FRlncRNAs

According to the FRlncRNAs related to prognosis, the hierarchical consensus clustering was used to perform the classification of TCGA cohort (20). To obtain robust classification, we adopted an unsupervised consensus approach implemented in the R package “Consensus Cluster Plus” (21). Moreover, the relative change in area under the cumulative distribution function (CDF) curve was employed to determine the optimal number of clusters, k, which was further verified by the total within sum of squares (WSS) and the gap statistics. The difference of survival probability and clinical information (age, stage, T stage, N stage, and M stage) between clusters were investigated.

### Evaluation of the Correlation With Immune Features

Inspired by the success of immunotherapy in the patients with BC in recent years (22), we further explored whether there was an immunological explanation for the survival differences between the clusters. Set PD-L1 gene as the strongest example, we carried out Pearson's correlation coefficient to test the co-expression and correlation between the hub gene and the prognostic FRlncRNAs in tumor tissues. Besides, ESTIMATE algorithm was performed to calculate the immune and stromal scores to quantify the presence of stromal cells and the infiltration of immune cells in tumor samples. To observe the differences of immune cells among clusters in the tumor microenvironment in a more detailed way, CIBERSORT, a gene expression-based deconvolution algorithm to describe the cell constitution of tissues (23), was performed to intuitively display the distribution of immune cells, which was showed in the violin plot generated by the vioplot package.

### Gene Set Enrichment Analysis (GSEA) Between Clusters

Gene Set Enrichment Analysis determines whether the predetermined gene sets have statistically significant differences between the two biological states in a computational method (24). In view of the consensus clustering, we conducted GSEA analysis in clusters with the aim of mining survival differences. By adjusting the *p*-value, the enrichment pathway for each phenotype was classified *via* the normalized enrichment score (NES). An NES >1 and false discovery rate (FDR) < 0.05 denoted statistical significance.

### Construction and Validation of the Prediction Models

Based on the results of univariate Cox regression analysis, the least absolute shrinkage and selection operator (LASSO) regression was applied to select the optimal survival-related FRlncRNAs, which were involved in the final modeling. According to the coefficients derived from LASSO regression and expression levels of FRlncRNAs included in final models, the prognostic risk score formula was constructed as follows:


$$\begin{array}{l} risk\;score=\sum_{n=1}^{i}\left(\beta_{n}*expression\;of\;gene_{n}\right) \end{array}$$

where β is the regression coefficient.

We randomly divided the patients with BC from TCGA into two groups according to the ratio of 1:1, one group as the training set and the other group as the validation set. In the training set, we calculated the risk scores of the patients with BC and classified these patients into the high-risk group and the low-risk group on the basis of the median risk score as the threshold. The Kaplan–Meier (K–M) survival analysis was used to prove whether there was a survival difference between the two groups. The receiver operator characteristic (ROC) curve was built by using the survival ROC package to assess the efficiency of the prognostic model. In the test group, the same processes were performed to validate the prognostic model of this group. Independent cohort validation is important for prognostic signatures. In the current study, the GSE69031 cohort was used to validate our OS signature (25). The expression data of the genes included in the final signature were obtained and substituted into the equation for risk score calculation. All patients in this cohort were stratified into low- or high-risk groups. The prediction accuracy of signature in the independent validation cohort was evaluated by ROC curve and K–M survival analyses.

### Identification of the Independence of Risk Score Prognostic Model

The clinical information, such as age and stage, was integrated to testify the independence of the prognostic model with the combination of risk score. For that, the univariate and multivariate Cox regression analyses were performed to verify the independence of the prognostic model in the training cohort and test cohort, respectively.

### Validation of the Risk Score Prognostic Model Between Different Subgroups

Through stratification of clinical data, K–M curves were drawn, respectively to study whether the genetic risk scores were applicable to patients in different groups. Specifically, we divided patients into the two categories based on age >65 and age <65, T1-2 and T3-4, N0 and N1–3, M0 and M1, Stage I–II and Stage III–IV, respectively, and calculate the difference in survival curves between the high-risk and low-risk patients in each category, so as to expand the applicability of risk scores.

### Comprehensive Analysis of the Differences Between High- and Low-Risk Groups

We enrolled all eligible patients and divided them into the high-risk and low-risk groups according to the calculation above. The clinical information (age, stage, T stage, N stage, and M stage), immune score, and clusters were integrated to exhibit the differences between high-risk and low-risk groups. More importantly, we also considered the expression differences of the survival-related FRlncRNAs involved in the final modeling, hoping to provide a theoretical basis for finding new therapeutic targets for BC.

## Results

### The LncRNAs Associated With Ferroptosis Genes

Through the co-expression analysis, we sorted out the 63 FRLncRNAs, and visualized the relationship by co-expression network (Figure 1). In the Figure 1, the red nodes represent the ferroptosis-related genes, and the blue nodes represent LncRNAs co-expressed with ferroptosis-related genes. These LncRNAs were used as FRlncRNAs for the subsequent analyses.

**Figure 1:** Co-expression network analysis on target LncRNAs related to ferroptosis-related genes. The red node represents the ferroptosis-related genes and the blue node represents the LncRNA coexpressed with the ferroptosis-related genes.

### Identification of the FRlncRNAs Related to Prognosis

To explore the influence of FRlncRNAs on the prognosis of patients with BC, the univariate Cox regression analysis was used to preliminarily determine 31 FRlncRNAs related to the prognosis, which were visualized by forest map (Figure 2). If the hazard ratio (HR) >1, the higher the expression level, the higher the risk of patients. On the contrary, HR < 1 means that the higher the expression level, the lower the risk of patients. Further, the differential analysis was employed to exhibit the expression level of 31 prognosis-related FRlncRNAs between the normal tissues and tumor tissues. LINC00702, AC121247.2, HSD11B1-AS1, NR4A1AS, AC011472.4, LIPE-AS1, etc., were lower expressed in tumor tissues, conversely, AP001434.1, LINC02257, LINC01655, LINC01614, AF015262.1, LMNTD2-AS1, etc., were highly expressed in tumor tissues (Figure 3).

**Figure 2:** Univariate Cox regression analysis of the FRLncRNAs related to prognosis. The red and green boxes represent risk factors or protective factors, respectively.

**Figure 3:** The heatmap shows the differential expression of the prognostic between normal and tumor tissues. ^*^P < 0.05, ^**^P < 0.01, ^***^P < 0.001.

### FRlncRNAs-Based Clusters Associated With Prognosis

Our study confirmed that some FRlncRNAs were related to the prognosis of patients, and were expressed in a heterogeneous manner among tumor patients. In order to better understand the intertumoral heterogeneity of BC, we conducted an unsupervised consensus analysis to explore the influence of FRlncRNAs on the occurrence and development of BC from multiple perspectives. Using the similarities in the expression of prognosis-related FRlncRNAs, we choose the value of *k* = 2 as optimal selection (Figures 4A,B). Consequently, the two clusters of samples were determined as follow: C1 (*n* = 726, 80.8%) and C2 (*n* = 172, 19.2%). We then applied K–M curves to compare the differences in survival between different clusters and found that C1 tended to carry a good prognosis (Figure 4C). Next, we researched whether there was a correlation between the clinical data and clusters (Figure 4D). It was obvious that the expressions of FRlncRNAs in the upper right corner of heatmap were upregulated in C2, with a more red color, such as AP001434.1, LINC02257, LINC01655, LINC01614, and AF015262.1. More interestingly, we noticed that most of these FRlncRNAs upregulated in C2 with poor prognosis were also upregulated in tumor tissue, suggesting that these FRlncRNAs may act as tumor promoters to accelerate tumor migration and progression. At the same time, we could also compare whether there were differences in clinical traits in different clusters. Figure 4D shows no significance in the clinical parameters indicating no differences between these characteristics in the various clusters.

**Figure 4:** Hierarchical consensus clustering based on the prognostic FRLncRNAs. **(A)** Consensus clustering analysis identification of two clusters (*n* = 896); **(B)** Cumulative distribution function (CDF) for *k* = 2–9; **(C)** Kaplan–Meier (K–M) curves for the 896 patients breast cancer (BC) stratified by cluster; **(D)** Heatmap on the prognostic FRLncRNAs ordered by clusters. The association with clusters, survival probability, and clinical information (age, stage, T stage, N stage, and M stage) were investigated.

### FRlncRNAs-Based Prognostic Differences Significantly Associated With Immune Features

To investigate the correlation of FRlncRNAs with immune features, we conducted further analysis from the perspective of immunology. The correlation analysis was performed to explore the relationship between prognosis-related FRlncRNAs and PD-L1 gene (Figure 5). The result implies that PD-L1 was significantly associated with some FRlncRNAs, such as LINC02328, LINC01871, LMNTD2-AS1, LINC00702, LINC02384, AP001434.1, TRG-AS1, LIPE-AS1, HSD11B1-AS1, USP30-AS1, LINC02446, AC099329.2, PRKAR1B-AS1, and LINC02084. Furthermore, we investigated the differences of immune microenvironment between the clusters. Intriguingly, we found that there was no difference in immune cells between C1 and C2 (Figure 6A), whereas C2 was associated with higher stromal scores compared with C1 (Figure 6B). Furthermore, violin plot analysis showed that the levels of cell infiltration (Figure 6C), such as B cells naïve, plasma cells, T cells CD8, T cells CD4 memory activated, T cells follicular helper, natural killer (NK) cells activated, monocytes, macrophages M1, dendritic cells resting, and neutrophils were higher in C1 than in C2, whereas the levels of macrophages M0 and macrophages M2 were lower in C1 than in C2. Collectively, the turbulent changes of immune cells in the tumor immune microenvironment may support the conclusion that C2 had a poor prognosis to some extent.

**Figure 5:** Correlation analysis between PD-L1 gene and the prognostic FRLncRNAs. Blue is a negative correlation, red is a positive correlation, and if there is an asterisk in the grid between two genes, they are significantly correlated.

**Figure 6:** Evaluation of the correlation with immune features between clusters. **(A)** Immune score between clusters; **(B)** Stromal score between clusters; **(C)** The violin plot of comparison of 22 types of immune cells between clusters.

### The Differential Biological States in Clusters Identified by GSEA Analysis

The explanation from the immune point of view made us understand the impact of target FRlncRNAs on tumor microenvironment more thoroughly. We further conducted GSEA analysis to explore the biological signal pathways with obvious differences between the clusters. Some metabolism-related pathways, in relation to “adipocytokine signaling pathway,” “linolenic acid metabolism,” “arachidonic acid metabolism,” “fatty acid metabolism,” “ether lipid metabolism,” and “glutathione metabolism” were significantly enriched in C1, among which the pathways related to lipid metabolism accounted for the majority (Figures 7A–F). In addition, we found that immune-associated pathway was enriched, such as “T cell receptor signaling pathway” and “TGF-beta signaling pathway” (Figures 7G,H). Besides, the enrichment of some carcinogenic pathways was also exposed, such as “pathway in cancer,” “apoptosis,” “cytosolic DNA sensing pathway,” and “base excision repair” (Figures 7I–L).

**Figure 7:** Gene Set Enrichment Analysis (GSEA) between the clusters **(A–L)**.

### Establishment and Validation of the Prognostic Signature in the Patients With BC

First, according to the ratio of 1:1, the patients with BC were randomly divided into a training set and a validation set, both of which included 448 patients with complete information, as described in the previous literature (26). Second, according to 31 prognostic FRlncRNAs calculated by univariate Cox regression analysis, we then performed LASSO regression analysis to pick out the optimal prognosis-related FRlncRNAs with nonzero coefficients (Figures 8A,B). Consequently, 12-FRLncRNA signature was determined. The formula of the final model was listed as follows: risk score = −0.250^*^expression of LINC01871+0.091^*^expression of LINC00393+1.058^*^ expression of AC121247.2-0.330^*^ expression of LINC02384-0.336^*^ expression of LIPE-AS1-0.072^*^ expression of HSD11B1-AS1+0.361^*^ expression of AC010655.2+0.018^*^ expression of LINC01419+0.051^*^ expression of PTPRD-AS1+0.137^*^ expression of AC099329.2+0.024^*^ expression of OTUD6B-AS1+0.157^*^ expression of LINC02266. We then calculated the risk scores and divided patients into high- and low-risk groups by the median risk score in the training set (Figure 9A). The relationships between the survival status and survival times of patients with BC ranked by risk scores were depicted in Figure 9B. In addition, a heatmap was plotted to show the expression profiles of 12 FRLncRNAs (Figure 9C). To study the relationship between the risk score and survival probability, K–M curves were carried out in Figure 9D. Patients in the high-risk group had a worse survival probability, whereas those in the low-risk group had a better survival probability. Furthermore, the ROC curve was plotted to verify the predictive ability of the models, whose AUC of the ROC curves was 0.693, revealing a positive prognostic ability (Figure 9E).

**Figure 8:** Selection of the optimal survival-related LncRNAs by LASSO Cox regression. **(A)** LASSO coefficient profiles of the candidate survival-related LncRNAs. A coefficient profile plot was produced against the log λ sequence. **(B)** Dotted vertical lines were drawn at the optimal values using the minimum criteria.

**Figure 9:** The 12-LncRNA signature in the training set. **(A)** The distribution of risk score; **(B)** the survival time and status of patients; **(C)** the bottom shows the heatmap of 12-LncRNA expression profile. Colors from red to green indicate decreasing expression level from high to low; **(D)** the K–M curves for high- and low-risk groups. Purple color represents the low-risk group, whereas red color represents the high-risk group; **(E)** receiver operator characteristic (ROC) curves for patients with BC in testing set. AUC, area under the curve.

To verify the results of the training set, we employed the same models on the patients in the testing set (Figure 10). The results showed that the high-risk patients showed significantly worse survival probability than the low-risk groups (Figure 10D), whose AUC of ROC was 0.655 (Figure 10E), which suggested that the prognostic model could satisfactorily predict the prognosis of patients with BC. In addition, the prognostic values of the risk score of patients with BC in the GSE69031 cohort were calculated. The results indicated that patients in the high-risk group showed a worse prognosis than the low-risk patients (Figure 10F). The AUC values of signature to predict the OS was 0.681 (Figure 10G). Generally, our signature showed satisfactory performance in the independent cohorts, which indicated that these signatures are robust prognostic biomarkers.

**Figure 10:** Testing for the 12-LncRNA signature. **(A)** The distribution of risk score; **(B)** the survival time and status of patients; **(C)** the bottom shows the heatmap of 12-LncRNA expression profile. Colors from red to green indicate decreasing the expression level from high to low; **(D)** the K–M curves for high- and low-risk groups. Purple color represents the low-risk group, whereas red color represents the high-risk group; **(E)** ROC curves for patients with BC in the testing set. **(F)** The K–M curves for the high- and low-risk groups in GSE69031 cohort. Purple color represents the low-risk group, whereas red color represents the high-risk group; **(G)** ROC curves for patients with BC in GSE69031 cohort. AUC, area under the curve.

### Exploration of Risk Score as an Independent Prognostic Factor

In view of the complexity of a variety of clinical factors, further univariate and multivariate Cox regression analyses were performed to explore the independence of risk scores (Figures 11A,B). Collectively, the risk score was an independent prognostic factor, independent of other clinical factors, in both the training and validation sets (*P* < 0.05). Generally, our research indicated that the patients with higher risk scores were a worse prognosis.

**Figure 11:** Identification of the independence of risk score prognostic model by the Cox regression analyses. **(A)** The univariate and multivariate Cox regression analyses of the risk score in the training cohort. **(B)** The univariate and multivariate Cox regression analyses of the risk score in the test cohort. The green boxes represent risk factors of the univariate Cox regression analysis and the red boxes represent risk factors of the multivariate Cox regression analysis.

### Model Validation of Clinical Grouping

First of all, we divided patients into the two categories based on age >65 and age <65, T1-2 and T3-4, N0 and N1-3, M0 and M1, Stage I-II, and Stage III-IV. By employing the same models, we plotted K–M survival curves for each subgroup (Figure 12). For example, in Figures 12C,D, patients with T stage at T1 and T2 showed statistically significant differences in their survival curves, and patients with T3 and T4 also showed statistically significant differences in their survival curves, indicating that the risk score was applicable to the patients with different T stages (*P* < 0.05). Similarly, in other grouping variables, such as age <65 and age> 65 (Figures 12A,B), in N0 and N1–3 patients (Figures 12E,F), in early and late-stage patients (Figures 12G,H), value of *P* < 0.05, indicating that the risk score of this gene was applicable to the different groups of patients. Nevertheless, among M0 and M1 stage patients, the difference was not statistically significant due to the small number of M1 stage patients, which required further data to verify. Overall, in the subgroup analyses, we confirmed that the high-risk patients were a worse prognosis than the low-risk patients in all subgroups (all *p* < 0.05).

**Figure 12:** Validation of the risk score prognostic model among the different clinical groups. **(A)** Age ≤65; **(B)** age >65; **(C)** T1-2; **(D)** T3-4; **(E)** N0; **(F)** N1–3; **(G)** stage I–II; **(H)** stage III–IV. The blue lines represent the low-risk groups, the red lines represent the high-risk groups.

### Relationships Between Risk Scores and Clinical Variables

Through a comprehensive analysis of the heatmap, we can easily distinguish the high-risk and low-risk FRLncRNAs (Figure 13). Specifically, LINC01871, LINC02384, LIPE-AS1, and HSD11B1-AS1 were highly expressed in low-risk groups, demonstrating that these FRLncRNAs were low-risk LncRNAs. On the contrary, LINC00393, AC121247.2, AC010655.2, LINC01419, PTPRD-AS1, AC099329.2, OTUD6B-AS1, and LINC02266 were highly expressed in the high-risk groups, demonstrating that these FRLncRNAs were high-risk LncRNAs. At the same time, we could also compare whether the clinical traits were different between the high- and low-risk groups. It could be seen that there were differences among the N stages, immune scores, and clusters (*P* < 0.05). More specifically, patients in the low-risk groups were more likely to be assigned to C1 and had a higher immune score, which were consistent with a better prognosis.

**Figure 13:** Comprehensive analysis of the differences between the high- and low-risk groups.

## Discussion

Breast cancer, as the most common female malignant tumor in the world, poses a serious threat to the life and health of women and has become a key global public health problem (1). To improve our understanding of pathogenesis and internal environmental changes in BC, we have made some efforts. Similar to a recent study (27), in this study, we downloaded and integrated the gene expression data of the transcriptome and the clinical information of patients with BC from TCGA dataset, starting with the downstream RNAs of the ferroptosis-related gene. However, unlike the previous study, unsupervised clustering analysis revealed that C1 tended to carry a better prognosis and held a higher infiltration level of immune cells than C2 in our study. Furthermore, GSEA analysis between C1 and C2 unveiled that C1 was enriched in lipid-metabolism-related pathway and immune-associated pathway, which was consistent with the outcomes of cluster analysis. Additionally, 12-FRLncRNA signature involved with LINC01871, LINC00393, AC121247.2, LINC02384, LIPE-AS1, HSD11B1-AS1, AC010655.2, LINC01419, PTPRD-AS1, AC099329.2, OTUD6B-AS1, and LINC02266 could accurately predict the prognosis of patients with BC, which was confirmed by the training set, validation set, and set from GEO database. Specially, PD-L1 was significantly associated with some FRLncRNAs. Combined with cluster analysis, prognostic model, and clinical characteristics, further analysis disclosure that patients in the low-risk groups were more likely to be assigned to C1 and had a higher immune score, which were in line with a better prognosis. These findings are based on ferroptosis, immune microenvironment, and prognosis of BC, which will provide theoretical guidance for the scientific application of ferroptosis and immunotherapy in BC.

According to the comprehensive analysis of 12-FRLncRNA signature, LINC01871, LINC02384, LIPE-AS1, and HSD11B1-AS1 were low-risk FRLncRNAs, whereas LINC00393, AC121247.2, AC010655.2, LINC01419, PTPRD-AS1, AC099329.2, OTUD6B-AS1, and LINC02266 were high-risk FRLncRNAs. For LINC01871, many studies have confirmed that it may be a protective factor of BC, promoting cancer cells death through many pathways and mechanisms, such as autophagy, which is consistent with our study results (7, 28, 29). Therefore, it can be speculated that IFNG co-expressed with LINC01871 was associated with promoting cell apoptosis by ferroptosis. As for LIPE-AS1, Zhang et al. (30) reported that overexpression of LIPE-AS1 in cervical cancer can promote cell proliferation, migration, epithelial mesenchymal transition (EMT), and inhibit cell apoptosis, which can be reversed by LIPE-AS1 knockdown or mir-195-5p/mitogen activated protein kinase (MAPK) signaling pathway activation.

Regarding LINC00393, Zhao et al. found that BC cells treated with CREBBP/EP300 bromodomain inhibitors can induce the downregulation of H3K27 acetylation level, along with downregulation of LINC00393 expression, which can inhibit the growth of BC cells, indicating it may therefore be a candidate for gene therapy approaches to BC (31). Besides, we also noticed that LINC00393 was coexpressed with SLC7A5, a protein in the amino acid transporter family, which is necessary for the growth of BC cells in a cell-dependent manner (32). In particular, SLC7A11 belonging to the same family is also closely associated with ferroptosis. Studies have shown that the deletion of SLC7A11 gene results in lipid peroxidation, which in turn leads to ferroptosis in some cells or tissues (33–36). In addition, LINC01419 has been repeatedly demonstrated to be upregulated in solid tumors and to promote proliferation and migration of malignant tumors through multiple pathways, such as PI3K/Akt signaling pathway, which is similar to our results and worthy of further study on the association of ferroptosis in BC (37–41). In addition, it has been reported that the overexpression of OTUD6B-AS1 makes hepatocellular carcinoma cells more aggressive through the GSKIP/Wnt/β-catenin signaling pathway (42). As for other FRLncRNAs, there are few studies on ferroptosis or malignant, and further studies are required.

More importantly, the findings of unsupervised clustering analysis showed that there were two different immune microenvironments. We found patients in the low-risk groups were more likely to be assigned to C1 and had a higher levels of immune cell infiltration, such as B cells naïve, plasma cells, T cells CD8, T cells CD4 memory activated, T cells follicular helper, NK cells activated, monocytes, macrophages M1, dendritic cells resting, and neutrophils, whereas the levels of macrophages M0 and macrophages M2 were higher in C2. In short, low-risk patients showed “hot tumor,” surrounded by immune-effector cells that are sensitive to immunotherapy, while high-risk patients showed “cold tumor,” which impair the effectiveness of immunotherapy (43). Morever, according to the results of GSEA analysis, we found that lipid-metabolism and oxidative stress pathways, such as “adipocytokine signaling pathway,” “linolenic acid metabolism,” “arachidonic acid metabolism,” “fatty acid metabolism,” “ether lipid metabolism,” and “glutathione metabolism,” were enriched in C1, as were immune-related pathways, such as “T cell receptor signaling pathway” and “TGFβ signaling pathway.” More interestingly, the studies have shown that when immunotherapy boosts the activity of T cells, it will increase the level of oxidized lipids in tumor cells, leading to the emergence of ferroptosis, which in turn will enhance the killing effect of immunotherapy on cancer (44, 45). Therefore, we can guess the following steps: C1, which is attributed to most low-risk patients, increases the level of lipid oxidation metabolism and induces ferroptosis; ferroptosis heats up the tumor immune microenvironment, activates immune-related pathways, wakes up immune cells, transforms “cold tumor” into “hot tumor,” upregulates the expression of PD-L1, enhancing the sensitivity of immunotherapy; the phenomenon of immune mobilization in turn promotes ferroptosis, forming a positive cycle. Collectively, for those tumors with insufficient induction of ferroptosis, the combination of ferroptosis sensitizers and immune checkpoint inhibitors to restore ferroptosis and improve the efficacy of immunotherapy may be a very promising combination therapy strategy. However, further studies are needed to determine the degree of induction and the degree of ferroptosis.

Our study comprehensively analyzed the relationships between ferroptosis, immune microenvironment, and prognosis of BC, which had a certain guiding significance for the designation of clinical immunotherapy combined strategy. However, there were certain limitations that existed in this study. First of all, we only used TCGA data to construct and verify our prognosis model, which lacked both revalidation from other public databases and validation from real-world data. Second, due to the lack of cell experiments or animal experiments to verify the expression of target FRLncRNAs or immune mechanisms, further identification and verification of therapeutic targets were needed. Third, only age and stage were included in the risk score independence analysis, which may increase the error of results due to the lack of clinical information.

## Conclusion

In summary, our study defined a novel 12-FRLncRNA signature associated with ferroptosis, which could accurately predict the prognosis in patients with BC. The comprehensive analysis of ferroptosis, immune microenvironment, and patient prognosis depends our understanding of the role of ferroptosis in shaping tumor microenvironment, which was of positive significance for basic research and clinical work in the future.

## Data Availability Statement

The datasets presented in this study can be found in online repositories. The names of the repository/repositories and accession number(s) can be found in the article/supplementary material.

## Author Contributions

ZX and SJ performed the data analysis. ZX, KF, and JM wrote the manuscript. JM, DT, and KF contributed to the manuscript revision. CY and DT contributed to the literature search and data extraction. ZX, SJ, and KF conceived and designed the study. All authors have read and approved the final version of the manuscript.

## Funding

This study was supported by the Ningxia Hui Autonomous Region Natural Science Foundation Project (Number: 2021AAC03523) and the Ningxia Hui Autonomous Region Key Research and Development Project (Number: 2021BEG03083).

## Conflict of Interest

The authors declare that the research was conducted in the absence of any commercial or financial relationships that could be construed as a potential conflict of interest.

## Publisher's Note

All claims expressed in this article are solely those of the authors and do not necessarily represent those of their affiliated organizations, or those of the publisher, the editors and the reviewers. Any product that may be evaluated in this article, or claim that may be made by its manufacturer, is not guaranteed or endorsed by the publisher.
